The article "The Empirical Analysis of Bitcoin Price Prediction Based on Deep Learning Integration Method" was published in 2022. Journal: Comput Intell Neurosci.

# The Empirical Analysis of Bitcoin Price Prediction Based on Deep Learning Integration Method

**DOI:** 10.1155/2022/1265837

**Published:** 2022-06-10

**Authors:** Shengao Zhang, Mengze Li, Chunxiao Yan

**Affiliations:** ^1^School of Public Administration, China University of Geosciences, Wuhan 430074, China; ^2^School of Public Finance and Taxation, Capital University of Economics and Business, Beijing 100070, China; ^3^School of Economics and Management, China University of Geosciences, Wuhan 430074, China

## Abstract

As a new type of electronic currency, bitcoin is more and more recognized and sought after by people, but its price fluctuation is more intense, the market has certain risks, and the price is difficult to be accurately predicted. The main purpose of this study is to use a deep learning integration method (SDAE-B) to predict the price of bitcoin. This method combines two technologies: one is an advanced deep neural network model, which is called stacking denoising autoencoders (SDAE). The SDAE method is used to simulate the nonlinear complex relationship between the bitcoin price and its influencing factors. The other is a powerful integration method called bootstrap aggregation (Bagging), which generates multiple datasets for training a set of basic models (SDAES). In the empirical study, this study compares the price sequence of bitcoin and selects the block size, hash rate, mining difficulty, number of transactions, market capitalization, Baidu and Google search volume, gold price, dollar index, and relevant major events as exogenous variables uses SDAE-B method to compare the price of bitcoin for prediction and uses the traditional machine learning method LSSVM and BP to compare the price of bitcoin for prediction. The prediction results are as follows: the MAPE of the SDAE-B prediction price is 0.016, the RMSE is 131.643, and the DA is 0.817. Compared with the other two methods, it has higher accuracy and lower error, and can well track the randomness and nonlinear characteristics of bitcoin price.

## 1. Introduction

Bitcoin is a decentralized, anonymous, exclusive ownership, and inflation-free currency [1]. Fry and Cheah [2] found that in view of the innovative characteristics of decentralization and traceability of bitcoin, bitcoin has attracted extensive attention from the media and investors. After the rise and fall of cryptocurrency prices in recent years, bitcoin is increasingly seen as an investment asset. Investors see bitcoin as a speculative investment, similar to the Internet stocks of the last century [3]. Bitcoin as a cryptocurrency, itself appears for a short time compared with the sovereign currency [4]. Unlike the sovereign currency, bitcoin is a decentralized digital currency without any government credit support, so the price of bitcoin is highly volatile. It produces much more volatility than sovereign currencies. Its price rose from zero value when it was established in 2009, to about $13 per bitcoin in January 2013, and then soared to about $20000 per bitcoin in December 2017. Since bitcoin started trading, its highly unstable nature has been plaguing investors, and it may be a bubble, threatening the stability of the financial system. Therefore, it is necessary to make a good prediction of the price of the special currency. The possibility of predicting the price trend of bitcoin is a practical problem. It not only affects a country's economic policy at the macro level but also strongly affects investors' decision to buy and sell investment instruments at the micro-level. Matkovskyy and Jalan [5] found that the accurate prediction of bitcoin price can not only provide decision support for investors but also provide reference for the government to formulate regulatory policies.

Equally noteworthy are the factors that influence bitcoin prices. In addition to the internal factors such as block size, hash rate, mining difficulty, trading volume, and market value of bitcoin, this study thinks that the factors should be more comprehensive: firstly, this study thinks that the Google and Baidu search index is an important factor affecting bitcoin because it is an important indicator to measure investors' attention and media hype and reflects the sentiment of the highly speculative cryptocurrency market [6]. Secondly, this study argues that the irrational factors such as major events and investor sentiment caused by economic policies will also affect the price of bitcoin [7]. Papadopoulos [8] shows that there is good interaction between bitcoin price and gold price. Dyhrberg [9] proved the similarity among bitcoin, gold, and the US dollar through the GARCH model. Therefore, this study takes the gold price and the dollar index as the influencing factors of bitcoin price. By selecting the above external factors, the problem of simplifying bitcoin price prediction is avoided.

The contribution of this study is as follows: compared with traditional financial asset price prediction, bitcoin price prediction is still in the early stage. Because bitcoin lacks seasonality, A. Greaves and Au [10] found that the machine learning model is applicable and useful. Similarly, Shah and Zhang [11] used Bayesian regression to predict the price change of bitcoin. At present, various popular machine learning algorithms such as SVM [12], RNN, LSTM, ARIMA [13], GA, and NARX [14] have also been applied to predict the price of bitcoin. Although the traditional machine learning model has obvious advantages in bitcoin price prediction, the imbalance and poor integrity of relevant data will lead to the problems of low accuracy, poor robustness, and easy to fall into the local optimum of deep network training. With the maturity of machine learning technology, deep learning has gradually become the mainstream of machine learning technology, and related algorithms and applications have also begun to flourish. And it shows strong ability in classification, feature extraction, and other nonlinear modeling tasks. A deep denoising self-coding network is a widely used network model in deep learning. With fewer data samples and suitable classification and recognition algorithms, it can obtain higher classification ability and has strong feature extraction ability and robustness. The unsupervised pretraining of self-coding networks can effectively extract the internal features of bitcoin data and reduce the loss of typical features to the greatest extent [13, 15]. Therefore, this study proposes a deep learning ensemble method (SDAE-B) to predict the price of bitcoin, which combines two technologies: one is the stacking denoising autoencoders (SDAE-B), which is used to simulate the nonlinear complex relationship between bitcoin price and its influencing factors. The other is a powerful integration method called bootstrapping, which generates multiple datasets for training a set of basic models (SDAES). Through the use of the SDAE-B method to compare the price of the special currency and get a good result.

The framework of this study is as follows: Section 2 introduces the methods proposed; Section 3 carries out empirical research and discusses the results; Section 4 gives the conclusion and describes the main contributions of the study.

## 2. Materials and Methods

### 2.1. Deep Learning Integration Method (SDAE-B)

Stacking denoising autoencoders (SDAE) [16] is a popular DNN model. The results show that it has higher prediction accuracy in a series of classification problems than competitive machine learning models such as stacked autoencoders (SAE) and deep belief networks (DBN). SDAE is constructed by stacking several denoising autoencoders (DAEs), which is a special neural network structure. To illustrate SDAE, the autoencoder (AE) and the DAE are introduced.

#### 2.1.1. Autoencoder (AE)

Autoencoder(AE) is a single hidden layer neural network with equal input and output sizes. Firstly, an input vector *x* ∈ [0,1]^*d*^ is mapped to a hidden representation *y* ∈ [0,1]^*d*′^ by a deterministic function:

(1) $$\begin{array}{c} y=f_{\theta }\left(x\right)=\phi_{f}\left(Wx+b\right). \end{array}$$

*F*(*x*) parametrization is *θ*={*W*, *b*}, *W* is a weight matrix of *d*′ × *d*, *b* is a bias vector, and *ϕ*_*f*_(·) is a nonlinear activation function. Then, *y* in the input space maps the return *z* ∈ [0,1]^*d*^ as the following equation:

(2) $$\begin{array}{c} z=g_{\theta^{\prime }}\left(y\right)=\phi_{g}\left(W{}^{\prime }y+b\right). \end{array}$$

With *θ*′={*W*′, *b*′}. Therefore, each training *x*^(*i*)^ is mapped to the corresponding *y*^(*i*)^ and reconstruction *z*^(*i*)^. The model parameters are optimized to minimize the average reconstruction error.

(3) $$\begin{array}{c} \theta^{*},\theta^{\prime *}=\arg_{\theta ,\theta {}^{\prime }}\min\frac{1}{n}\sum_{i=1}^{n}L\left(x^{\left(i\right)},z^{\left(i\right)}\right)=\arg_{\theta ,\theta {}^{\prime }}\min\frac{1}{n}\sum_{i=1}^{n}L\left(x^{\left(i\right)},g_{\theta }\left(f_{\theta }\left(x^{\left(i\right)}\right)\right)\right), \end{array}$$

where *L* is the loss function, which can be the traditional square error:

(4) $$\begin{array}{c} L\left(x,z\right)={\left\|x-z\right\|}^{2}, \end{array}$$

or reconstruction fork:

(5) $$\begin{array}{c} L_{H}\left(x,z\right)=H\left(B_{x}•B_{z}\right)=-\sum_{k=1}^{d}\left[x_{k}\log z_{k}+\left(1-x_{k}\right)\log\left(1-z_{k}\right)\right]. \end{array}$$

Vincent et al. [17] believed that the autoencoder (AE) is a self-monitoring algorithm, not an unsupervised algorithm. It does not need to mark the training samples, and its label is generated from the input data. Therefore, it is easy to train a specific encoder for the input of the specified class without any new work. The autoencoder (AE) is data-related and can only compares data similar to training data. For example, the automatic encoder trained with face has poor performance in compressing other pictures, such as trees, because the features it learns are related to the face.

#### 2.1.2. Denoising Autoencoder (DAE)

Based on the autoencoder (AE), the denoising autoencoders (DAE) adds noise to the input data of the input layer to prevent the overfitting problem, which improves the robustness of the learned encoder. The core idea of DAE is to reconstruct a purified input from a corrupted version. First, the corrupted original input data *x* is randomly mapped $\tilde{x}∼q_{D}\left(\tilde{x}|x\right)$ to $\tilde{x}$. Then input the noisy model $\tilde{x}$ and get *y* by $y=f_{\theta }\left(\tilde{x}\right)=\phi \left(W\tilde{x}+b\right)$ mapping. Finally, the pair is mapped *z*=*g*_*θ*′_(*y*) back to *z*. For the training set, the best parameters *θ* and *θ*′ are obtained by minimizing the average reconstruction error between *z* and undamaged input *x*. The process is shown in Figure 1.

#### 2.1.3. Stacking Denoising Autoencoders (SDAE)

The idea of stacking denoising autoencoders (SDAE) is to stack multiple DAEs together to form a deep architecture. Only when the training is complete, the input will be added with noise. It follows layer-by-layer greedy training [18]: each layer of the self-coding layer carries out unsupervised training independently to minimize the error between the input (the input is the hidden layer output of the previous layer) and the reconstruction result. After the former *k* layer is trained, the *K* + 1 layer can be trained, because the output of the *k* layer has been calculated by forwarding propagation, and then the output of the *k* layer is used as the input of *K* + 1 to train *K* + 1 layer.

Specifically, the first DAE uses the training set as the input for independent training and learns through *f*_*θ*_^(1)^ mapping function. Then the second DAE uses the hidden representation *y* of the first DAE as input to train and learn by *f*_*θ*_^(2)^ mapping function. All DAEs can train independently according to the same procedure. An independently supervised learning algorithm (such as FNN) is added to the structure, which uses the hidden representation of the last DAE as input. Finally, establish SDAE. Once the SDAE training is completed, its high-level characteristics can be used as the input of the traditional monitoring algorithm. Besides, the parameters of each layer of SDAE can be adjusted synchronously by gradient descent and other training algorithms. The process is shown in Figure 2.

#### 2.1.4. Bagging

Bagging [19] is the abbreviation of bootstrap aggregating. It is a powerful integrated learning algorithm, which can be used for tasks such as two classifications, multiclassification, and regression. Its principle is to give a data set containing *m* samples, first, take a sample randomly and put it into the sampling set, and then put the sample back, so that the sample will still have the chance to be selected in the next sampling. So, after *M* times of sampling, we can get a data set with the same data amount of *m* from the original data set. Simply speaking, there are put back samples in the statistics and each sample. The probability of samples being taken is the same, which is one of the total samples.

Only when the basic learning algorithm is unstable, bagging can generate different basic models, which can be regarded as a method to improve the prediction accuracy by using this instability. The neural network model is unstable due to the random initialization process of weights, while the bagging neural network has strong robustness. It has been successfully applied in the field of finance and economy [20–22]. For these reasons, bagging can be used to construct an integration based on SDAES.

#### 2.1.5. Multivariate Forecasting

Different from the time series model, the multivariate model not only considers the autoregressive effect of target series but also considers the influence of exogenous variables on the target series. The multivariate model as a simple but very important method in the process of statistical analysis, it has been widely used in prediction in different fields. For example, Rombouts et al. [23] applied it in the field of option pricing. In recent years, scholars have applied multivariate model and deep learning technology to the field of prediction [24]. The results show that the multivariate model outperforms the univariate model for forecasting. It can be formalized as a function to simulate the relationship between dependent variables and independent variables:

(6) $$\begin{array}{c} y\left(t+h\right)=f\left(s\left(y\right),s\left(x_{1}\right),\ldots ,s\left(x_{C}\right)\right), \end{array}$$

where *y*(*t*+*h*) is the value of the dependent variable in (*t*+*h*) and *s*(*x*)=*x*(*t*), *x*(*t* − 1),…, *x*(*t* − *l*_*x*_+1) is a set of past values of exogenous variable *x* with a total of *l*_*x*_. Therefore, the input quantity is *m*=∑*l*_*y*_+*l*_*x*_1__+*l*_*x*_2__+⋯+*l*_*x*_*C*__.

#### 2.1.6. The Overall Process of SDAE-B Approach

The main idea of the hybrid model is as follows. The deep learning model SDAE is used to extract useful information from the selected data and generate prediction. The powerful integration method bagging is used to combine the strength of multiple SDAEs to improve the prediction accuracy, so as to generate an integrated model with better performance.

SDAE-B forecasts bitcoin prices based on the following five steps.  Figure 3 shows the flow chart of the whole process:

1. Data preprocessing: transform the original data into training samples and test samples.
2. Generate multiple training sets: generate K sample sets of training samples through the bootstrapping algorithm.
3. Training: each group of training samples trained K SDAE models, respectively.
4. Prediction: use SDAE models of K training to generate K predictions.
5. Result summary: take the average of K predicted values as the final result.

## 3. Results and Discussion

In this section, we compare the prediction ability of LSSVM and BP with that of SDAE-B. Firstly, the data description is given. Secondly, the model evaluation criteria are given. Then LSSVM, BP, and SDAE-B are used to compare the price of the special currency for prediction. Finally, the comparison results are given and analyzed.

### 3.1. Datasets

In this study, the data of bitcoin block size, hash rate, mining difficulty, number of transactions, and market capitalization are from Data.Bitcoinity.Org, Blockchain.com, and CoinMarketCAP. Baidu and Google search volume, respectively, come from Baidu Index and Google Trends. Relevant major events come from the review of the 11th anniversary of bitcoin by the blockchain media “Daily Star.” Gold prices come from GOLDHUB. Dollar index from Investing.com. The data is from November 29, 2014, to March 30, 2020. This study selects nine indicators of bitcoin, including block size, hash rate, mining difficulty, trading volume, market value, Baidu, and Google search volume, gold price, dollar index, relevant major events (Table 1) as independent variables, and bitcoin price (trend as shown in Figure 4) as dependent variables to build the model, as shown in Table 2.

The reasons for choosing these variables are as follows. First, they are closely related to bitcoin prices. Secondly, the relationship between bitcoin price series and these factors is noisy, fluctuating, and nonlinear, but any of them may provide useful information about bitcoin price trends at a certain point in time. Therefore, we can extract more information through as many variables as possible. Finally, as a deep neural network model, SDAE has a very powerful function in high-dimensional data modeling. Using these variables, we can make full use of the advantages of SDAE to create an ideal environment for the modeling of the bitcoin price series.

Different from previous studies, except for the internal factors such as block size, hash rate, mining difficulty, trading volume, and market value of bitcoin, this study increases Baidu and Google search volume, gold price, dollar index, and relevant major events.

These variables are selected to model the price series of bitcoin for the following reasons: first, they are closely related to bitcoin prices and represent different drivers of bitcoin prices. Secondly, the relationship between bitcoin price series and these factors is noisy, unstable, and nonlinear, but any of them may provide useful information about the movement of bitcoin price at a certain time. Therefore, we can extract more information by including as many variables as possible. Finally, a large number of variables can be used to provide relatively complete bitcoin price change information.

To model, this study divides the data into two parts: the training sample contains the first 80% of the observation values of all series, and the rest is the test sample. For model training, bitcoin price and exogenous variables are preprocessed by the normalization method.

### 3.2. Model Evaluation Index

To evaluate the prediction performance of the model from different perspectives (i.e., direction prediction and level prediction), three frequently used indicators in recent years include direction accuracy (DA), mean absolute error (MAPE), and mean square root error (RMSE):

(7) $$\begin{array}{c} DA=\frac{1}{N}\sum_{t=1}^{N}a\left(t\right)\times 100\%,\\ MAPE=\frac{1}{N}\sum_{t=1}^{N}\left|\frac{y\left(t\right)-\hat{y}\left(t\right)}{y\left(t\right)}\right|,\\ RMSE=\sqrt{\frac{1}{N}\sum_{t=1}^{N}{\left(y\left(t\right)-\hat{y}\left(t\right)\right)}^{2}}, \end{array}$$

where *y*(*t*) and $\hat{y}\left(t\right)$ represent true value and prediction respectively when $\left(y\left(t+1\right)-y\left(t\right)\right)\left(\hat{y}\left(t+1\right)-y\left(t\right)\right)\geq 0,\;a\left(t\right)=1$; otherwise, *a*(*t*)=0. N is the size of the forecast data.

### 3.3. Parameter Settings

SDAE model is a three-layer hidden neural layer network model. It stacks two DAEs and a supervised FNN on top of the architecture. According to the size of the feature space, set the number of nodes in the first to third hidden layers to 200, 100, and 10. Based on the trial and error method, the number of epochs for DAEs unsupervised pretraining, FNN supervised pretraining, and global fine tuning are all set to 500. The noise type in DAEs is additive Gaussian noise. According to Vincent et al. [17], the noise ratio is 0.2. The numbers of *K* is set to 100. The choice of *K* number is actually a trade-off between computational complexity and accuracy. However, with the increase of *K*, the prediction error of SDAE-B quickly converges to a certain level, so it is not necessary to select a large number. The lagged order of all variables and bitcoin price in the multivariate prediction model is set to 1, i.e., to learn a function satisfying. Through this method, a short term nonlinear dependency can be learned between input/output data. The number of hidden layers of BP is 1, the network structure is [40, 20, 1] the activation function is sigmoid function, and the learning rate is 0.1. The Gaussian kernel function is selected as the kernel function of the LSSVM method. Matlab R2016a is used to perform all the computations in this study.

### 3.4. Bitcoin Price Forecast

With the help of MATLAB software, LSSVM, BP, and SDAE-B are used to compare the price of special currency for forecasting. The results are shown in (Table 3). Also, the research results are shown in Figures 5–7.

The results show that SDAE-B has higher direction accuracy (DA), lower mean absolute error (MAPE), and lower mean square root error (RMSE), and has better prediction performance than LSSVM and BP. The possible reasons are as follows:

1. When dealing with data with various features, many traditional machine learning algorithms have a weakness. They cannot extract and organize different information from the data. Since it may be a difficult task to build a model of the relationship between bitcoin price and many variables, traditional models may not be able to learn useful representations, resulting in poor out of sample predictions. Instead, SDAE-B has a deep architecture. It can learn useful information from features by extracting multiple levels of representation, to obtain better prediction ability when the sample data are insufficient.
2. The performance of the integrated model is more stable than the traditional single machine learning model, because the traditional single machine learning model excessively relies on the sample data, underestimates the variance, and causes overfitting. The integrated model can reduce overfitting or generalization errors.

## 4. Conclusions

At present, bitcoin is a good stored value and safe haven, which is the most important use of bitcoin by all those who recognize it. In the long run, with the continuous development of blockchain technology and the recognition of bitcoin by more and more countries, bitcoin is likely to become a national strategic reserve resource like gold. Although the price of bitcoin is of great significance to market practitioners, the theoretical research in this field is very limited. In this study, a deep learning integration method named the SDAE-B is utilized to predict the price of bitcoin. Aiming at the complex relationship between bitcoin price and various factors, this study proposes LSSVM, BP, and SDAE-B to predict bitcoin price. In the data selection, through the analysis of internal and external factors, the limitations of the previous bitcoin price prediction methods, which only consider the historical data of bitcoin price are overcome. In empirical research, the first step is to obtain data, and then do data processing and model training. Through the training results, we can get a bitcoin price prediction based on deep learning and get good results. The SDAE-B model is better than the LSSVM model and BP model, which have higher accuracy and lower error. It shows that this method can be used as a promising tool for bitcoin price prediction.

Nevertheless, this study think there is still room for improvement. As we all know, unconventional factors such as political risk and investor psychology also have a great influence on the price fluctuation of special currency, but how to quantify the influence of these factors is quite challenging. This study believes that better predictions can be generated by quantifying these factors and using the information they provide. Finally, the prediction results of the SDAE-B model proposed in this paper have a certain lag, and the correction of postphenomenon is also the focus of future research.

## Figures and Tables

**Figure 1:** The architecture of DAE.

**Figure 2:** The architecture of SDAE.

**Figure 3:** The prediction process of SDAE-B model.

**Figure 4:** Bitcoin price trend in recent five years.

**Figure 5:** Comparison of the true price of Bitcoin and predicted price based on SDAE-B model.

**Figure 6:** Comparison of the true price of Bitcoin and predicted price based on LSSVM model.

**Figure 7:** Comparison of the true price of Bitcoin and predicted price based on BP model.

**Table 1:** Features.

Future	Definition
Block size	The average block size in MB
Hash rate	The estimated number of tera hashes per second (trillions of hashes per second), the bitcoin network is performing
Mining difficulty	A relative measure of how difficult it is to find a new block. The difficulty is adjusted periodically as a function of how much hashing power has been deployed by the network of miners
Number of transactions	The number of transactions per day
Market capitalization	The total US dollar market value of bitcoin
Baidu and google search volume	The weighted volume for media coverage of the keyword “bitcoin”
Relevant major events	Major events in bitcoin from November 29, 2014, to March 31, 2020 (positive impact expressed as “1” and negative impact expressed as “−1”)
Gold price	XAU gold spot price in US dollars
Dollar index	An indicator that comprehensively reflects the exchange rate of the US dollar in the international foreign exchange market

**Table 2:** Summary statistics of features used for bitcoin price prediction.

Future	Count	Mean	Sd	Minimum	Maximum
Block size	1950	734528.0	189090.04	187483.7	998175.2
Hash rate	1950	3.24E + 18	3.86E + 18	9.98E + 15	1.81E + 19
Mining difficulty	1950	3.54E + 12	4.53E + 12	39457671307	1.66E + 13
Number of transactions	1950	238145.4	81220.36	59344	490644
Market capitalization	1950	70265662078	69380000349	2.53E + 10	3.23E + 11
Baidu and Google search volume	1950	594.84	296.41	232	2499
Major events	1950	0.09	0.84	−1	1
Gold price	1950	444.3	40.86	364.63	585.01
Dollar index	1950	96.08	2.88	87.98	103.61

**Table 3:** Forecast results.

Model	DA	MAPE	RMSE
LSSVM	0.658	0.106	272.152
BP	0.740	0.040	540.084
SDAE-B	0.817	0.016	131.643

## Data Availability

In this study, the data of bitcoin block size, hash rate, mining difficulty, number of transactions and market capitalization are from Data.Bitcoinity.Org, Blockchain.com, and CoinMarketCAP. Baidu and Google search volume, respectively, come from Baidu Index and Google Trends. Relevant major events come from the review of the 11th anniversary of bitcoin by the blockchain media “Daily Star.”. Gold prices come from GOLDHUB. Dollar index from Investing.com.
